# Solution for sports image classification using modified MobileNetV3 optimized by modified battle royal optimization algorithm

**DOI:** 10.1016/j.heliyon.2023.e21603

**Published:** 2023-10-31

**Authors:** Bing Wang, Asad Rezaei sofla

**Affiliations:** a School of Physical Education, Zhengzhou Normal University, ZhengZhou, HeNan, 450044, China; b Islamic Azad University, Tehran, Iran; c College of Technical Engineering, The Islamic University, Najaf, Iraq

**Keywords:** Sports image, Classification, Modified battle royal optimization algorithm, MobileNetV3

## Abstract

Sports image classification using image processing and machine vision is a growing area of research that involves the use of algorithms and techniques to identify and analyze objects in sports images and videos. This technology has a wide range of applications, including detecting illegal plays, analyzing team performance, and creating highlight reels. Additionally, it can provide valuable visual feedback during training and competition. In this paper, we propose a novel deep learning and optimization hybrid framework for sports image classification. Specifically, we use a modified version of the Battle Royal optimization algorithm as a feature selector to reduce the dimensionality of the images and achieve higher accuracy with only the essential features. We evaluate the proposed framework using sports images and demonstrate that our WOA-based framework outperforms other methods in terms of both classification accuracy and dimensionality reduction. Our results highlight the effectiveness of the proposed approach and its potential to improve sports image classification.

## 1 Introduction

### 1.1 Background

Massive amounts of multimedia material have been produced and sent across the internet during the last couple of decades [1]. The majority of the multimedia information that is available online is made up of sports footage. Sport is a significant component of many broadcast mediums, including live streaming services, television, internet, etc. Each day, lots of sports-related videos overwhelm data servers [2]. Due to the huge global viewership and possible economic benefits, sports video content analysis has received a lot of attention. Such a large amount of video information is difficult to manually annotate. Therefore, automated techniques for managing and analyzing sports video footage are needed [3].

While watching and browsing interactive databases, people are drawn to significant notions, hence indexing and semantic video content evaluation are becoming more and more important. The provision of user-relevant semantic information is the main objective of video content analysis and management [4]. Researchers have suggested several automatic and semi-automated methods for this aim, including crucial recognition, video summarizing, and shot categorization [2].

A significant phase of the expanding subfields of artificial intelligence is deep learning. Deep learning, is a new technique based on neural networks that can provide a high-accuracy classification based on the trained data [5]. The main feature of deep learning methods is that they don't need an extra feature extraction phase for the classification.

The goal of image classification is to recognize and describe the characteristics that appear in a picture in terms of the real object that these characteristics truly represent on the ground as a distinct gray level (or color) [6]. The most crucial aspect of digital image analysis is probably picture categorization. Since distinguishing between different objects is a difficult operation, picture classification has been a crucial task in the field of computer vision. The labeling of pictures into one of some predetermined classifications is referred to as image classification [7].

A particular image can be categorized into one of n possible classes. It might be time-consuming to manually review and categorize large numbers of images, thus it would be really helpful if we could completely automate this procedure using computer vision.

There have been several research studies on image classification applications for sports imagery. Because of their thorough examination and effective outcomes, classifiers include the Bayesian classifier [8], InceptionV3 [3], and convolutional neural network with DE algorithm [7].

### 1.2 Related works

Chen et al. [9] investigated the use of the CNN method to analyze port Sequence Images. This paper presents a novel algorithm combining single-frame and multi-frame detection techniques to enhance the detection rate of small targets while shortening the detection time. Additionally, an enhanced, multi-scale, residual network based on a traditional residual network is proposed. This network architecture grants convolution layers access to more input features from different scales and decreases the complexity of training. Finally, an ensemble learning strategy of relative majority voting is employed, bringing down the classification error rate of the network to 3.99 % on CIFAR-10, 3 % lower than the original residual neural network.

Hsu et al. [10] investigated the application of the Deep CNN method to classify Wearable Sports Activity. An innovative wearable sports activity classification system has been established with a deep learning-based classification algorithm to accurately recognize 10 sports activities. The system utilizes two inertial sensing modules worn on the wrist and ankle of athletes, and a deep convolutional neural network (CNN) to generate features from the spectrograms. Evaluations demonstrate that the system can recognize 10 sports activities with an accuracy rate of 99.30 %.

Russo et al. [11] utilized a combination of deep learning methods and transfer learning to investigate the categorization of sports videos. This research utilizes a combination of convolutional and recurrent neural networks to distinguish 15 distinct sports classes. Transfer learning is applied to the VGG-16 model, resulting in 94 % and 92 % accuracy when assessing 10 and 15 sports classes, respectively. These results apply to digital content archiving in broadcasting companies as well as recognizing human actions. The VGG-16 model was able to reach impressive test accuracies of 94 % and 92 % for 10 and 15 sports classes, respectively.

Minhas et al. [2] employed the AlexNet CNN method to classify field sports videos. This study offers an effective approach for classifying shots in field sports videos with the use of AlexNet CNN. It has five convolutional layers and three fully connected layers and was tested on cricket and soccer video datasets. It achieved an impressive accuracy of 94.07 %, outperforming the existing state-of-the-art shot classification techniques.

Guangyu et al. [12] utilized a neural network algorithm and transfer learning to implement an analysis of sports video intelligent segmentation technology. The emergence of information technology has generated an abundance of digital content, making the precise categorization of sports videos essential. Consequently, deep neural networks, convolutional neural networks, transfer learning, block brightness comparison coding, and block color histogram have been employed to facilitate this. Results have demonstrated that the sports video image classification approach based on a deep learning coding model is more efficient.

Liu et al. [13] utilized Motion Action Examination of a Basketball Sports Scene using Image Processing. This paper proposes an analysis method of motion action in basketball sports scenes based on the Spatial-Temporal Graph Convolutional Neural Network (STGCN) to address the issues of low accuracy and high time cost associated with manual recording and statistics. The proposed method utilizes a graph structure to model human body joints and limbs, an STGCN structure to model posture action, and a combination of classification and transfer learning for the recognition of motion fuzzy posture. The effectiveness of the proposed method is demonstrated by analyzing the motion action using OpenCV with an average recognition accuracy of over 75 %, thus indicating its potential practical application.

### 1.3 Motivation and contribution

To enhance the effectiveness of video detection for sports wrong actions under wireless networks, a remote video detection algorithm was proposed by Liu and Yang [14] that extracted key frames and established a real-time video transmission model based on wireless networks. The deterministic constrained nonlinear optimization method was used to estimate motion parameters, and the aggregated channel feature method was used to identify targets in the video sequence. The support vector machine was used as a classifier of sports actions to recognize wrong actions. A multi-scale space of moving images was constructed, and a multi-layer box filter was used to simulate Gaussian convolution. The results showed that the proposed algorithm achieved a fidelity rate of over 90.3 % and a compression rate of over 80 %, with only one key point omitted. The experimental results demonstrate the high fidelity and compression rates of the proposed algorithm and verify its effectiveness in detecting sports wrong actions remotely.

The majority of the algorithms for classifying sports images that have been given, meanwhile, have drawbacks that reduce classification precision. It has been observed that these restrictions are caused by either the method used to extract the features or the method used to decrease the number of characteristics that were picked. This inspired us to offer a different sports picture categorization technique.

The proposed research work adds a novel approach to sports image classification using a hybrid deep learning and optimization framework. Specifically, the modified version of the Battle Royal optimization algorithm is used as a feature selector to reduce the dimensionality of images and achieve better accuracy by selecting essential features. Compared to existing methods in the literature, this approach offers several advantages. Firstly, it provides improved accuracy rates for sports image classification tasks. Secondly, it reduces dimensionality without sacrificing performance, which can lead to faster processing times and more efficient use of computational resources. Finally, it has potential applications in various areas such as screening illegal plays or creating highlight reels from games. Overall, this research work introduces an innovative method that combines deep learning techniques with optimization algorithms to improve sports image classification accuracy while reducing computational complexity. This makes it a valuable contribution to the field of machine vision and artificial intelligence applied within the domain of sports analysis.

## 2 Materials and methods

The main purpose of this research is to propose a MobileNetV3 and optimization hybrid framework for sports image classification. To achieve this, we have developed a methodology that utilizes a modified version of the Battle Royal optimization algorithm as a feature selector to reduce the dimensionality of the images and improve the accuracy of the classification. The proposed framework has been tested on a dataset of sports images, and the results have shown that it outperforms other methods in terms of both classification accuracy and dimensionality reduction. In this section, we will describe the materials used in this study, as well as the methods and techniques employed to analyze and process the data. Specifically, we will provide details on the image dataset, the deep learning architecture used, the optimization algorithm employed, and the evaluation metrics used to assess the performance of the proposed framework. The materials and methods section will also describe the experimental setup used to validate the results and provide insights into the strengths and limitations of the proposed framework. Here is a pseudocode for the proposed approach:

**Table:** 

Algorithm 1
(1) Load and preprocess the dataset of sports images. (2) Define the MobileNetV3 deep learning model architecture. (3) Initialize the modified Battle Royale optimization algorithm. (4) Train the MobileNetV3 model using the training set of the dataset. (5) Select the most important features of the images using the Battle Royale optimization algorithm. (6) Train the MobileNetV3 model using only the selected features. (7) Test the performance of the model using the test set of the dataset. (8) Compare the performance of the proposed method with other state-of-the-art methods, including InceptionV3, Bayesian classifier, and convolutional neural network. (9) Evaluate the results and calculate the accuracy of the proposed method across all sports categories. (10) Analyze the accuracy rates of the proposed method in specific sports categories, such as volleyball, badminton, and tennis. (11) Incorporate temporal information into the framework for activity analysis and video searches.

### 2.1 MobileNetV3

Deep learning is a form of artificial intelligence that uses machines instead of humans. Our brains are made up of nerve fibers that are connected and process information based on the inputs we receive. Deep learning works similarly, using a deep neural network to act like the human brain. With an increasing number of layers and neurons in each hidden layer, the model complexity grows. When these neural networks have more than three input and output layers, they are referred to as deep neural networks, which are known as deep learning. It is thought that complex problems in prediction and classification can be simplified by using these deep neural networks.

Deep learning is a process that converts input into output. Deep neural networks discover the correlation between input and output data. The “depth” of the neural network implies that these networks are multi-layered. The layers of the neural network are composed of nodes, which are analogous to the human brain in that they perform calculations [15]. In a node, the input data is multiplied by a weight, with higher weights having a stronger influence on the data; afterward, the sum of all data multiplied by their respective weights is calculated. Finally, to reach an output, the resulting total undergoes an activation function and produces an output.

Deep learning is the process of learning through neural networks that contain numerous hidden layers. For example, deep learning divides images into separate layers, similar to how the human brain works and brain cells are sensitive to masses. This allows them to recognize the entire image and process it accordingly.

Convolutional Neural Networks (CNNs) are a type of deep neural network that has become extremely useful for recognizing visuals, such as objects, faces, and traffic signs. They're most commonly utilized in deep learning for image and video recognition, image classification, medical imaging analysis, and language processing. CNNs are also integral in the development of self-driving cars and robots.

Utilizing convolutional neural networks, deep learning provides an invaluable tool for analyzing visual images. From image and video recognition to medical image analysis and language processing, the applications for this deep neural network are vast and varied.

Since the advent of the AlexNet convolutional network in computer vision, convolutional neural networks have gained immense popularity. Computer vision has had a massive impact on various fields. Despite the complexity of these networks, attempts have been made to decrease the total number of parameters while still retaining a high level of accuracy in design. Ultimately, accuracy was the primary focus in the development of these networks.

Since the advent of the AlexNet convolutional network in computer vision, convolutional neural networks have gained immense popularity. Computer vision has had a massive impact on various fields. Despite the complexity of these networks, attempts have been made to decrease the total number of parameters while still retaining a high level of accuracy in design. Ultimately, accuracy was the primary focus in the development of these networks.

The necessity of high-speed, lightweight networks with applications in robotics, minicomputer boards, and mobile phones was evident. Subsequently, this gave rise to a new class of light convolutional networks, featuring low parameters and high execution speed while maintaining satisfactory accuracy. A major example of such a network is MobileNet, which was designed by Google researchers for creating efficient networks that are lightweight, fast, and accurate. Previous research on the topic can be found in the related works section of the principal article.

MobileNetV3 is a convolutional neural network designed to be optimized for use on mobile phone CPUs using a hardware-aware network architecture search (NAS) combined with the NetAdapt algorithm, as well as further improved through novel architectural enhancements. The MobileNetV3 architecture integrates several building blocks and components from previous versions, as presented in Fig. (1).

**Fig. 1:** MobileNetV3 architecture.

Moreover, a novel type of nonlinearity, known as the hard swish ($h_{swish}$), is employed to reduce model complexity and the number of training parameters. This nonlinearity is defined in the Equation [1,2].

(1) $$h_{swish}=x.\gamma \left(x\right)$$

(2) $$\gamma \left(x\right)=\frac{ReLU6\left(x+3\right)}{6}$$

The variable γ(x) symbolizes the segmented hard analog function.

Fig. (1) demonstrates that the MobileNetV3 block is equipped with an innovative core building block termed the inverted residual block, which is comprised of a depth-wise separate convolution block and a squeeze-and-excitation block. This inverted residual block draws inspiration from bottleneck blocks, utilizing an inverted residual connection to link the input and output features on the same channels, thereby providing significantly enhanced feature representation without consuming excessive memory.

A depth-wise separable convolution utilizes a depth-wise convolutional kernel applied to the channels and a 1 × 1 pointwise convolutional kernel with a BN (batch normalization layer) and either the ReLU or h-swish activation functions. This form of convolution is used to modify conventional convolution blocks and decrease the capacity of the model. Additionally, a SE (squeeze-and-excitation) block is integrated to focus more on pertinent features for each channel during training.

### 2.2 Modified battle royal optimization algorithm (MBRA)

#### 2.2.1 Battle royal game theory

Battle Royale is inspired by a Japanese movie and the players of this game compete with each other. Players prevent themselves from being eliminated in the game by exploring the game area. The number of people who can play in Battle Royale is a minimum of two and a maximum of five. Considering that the players in this game are exposed to mayhem, the resources, and potency of each of them are the same [5,[16], [17], [18], [19]]. The game starts with the random distribution of players in the game space. The game starts with the random dispensation of players in the game region. The limited space in the game is called the secure zone and this area is gradually reduced. When the player goes out of the designated area, he is called a harmed or excluded player. In this game, some implements can help players to stay in the game. Ring of Elysium, Apex Legends, PUBG, Counter-stroke: Global Offensive, and Call of Duty: Warzone, are examples of Battle Royale games. In the mentioned games, players are given a chance to rejuvenate and in some cases, players are awarded for remaining in the game. These characteristics have been utilized to design the optimization algorithm. Finally, the winner of the game is a player or a team. Specifying the map related to the game area is the responsibility of the players [4,20]. Sanhok is one of the well-known maps in PUBG. Players in the secure region attempt to be close to each other so as not to receive the damaged card. The map of the safe zone is marked with a special color. Players in the secure region attempt to be close to each other so as not to receive the damaged card. The plan of the safe zone is marked with a special color. As the game space shrinks, the new safe zone is shown with a different color. To continue and stay in the game, players eliminate or kill their competitors. This mode is called death match. In this game, the winner will be the one who eliminates more individuals. Likewise, throughout the game, the player who is eliminated or killed can become visible in the game area haphazardly.

#### 2.2.2 Optimization algorithm of battle royal

Sometimes at the beginning of the game, players enter the game with an airplane or a parachute. At the beginning of the algorithm, a population is considered as a player that is scattered in the search space. Every one of the players attacks the opponent with a gun to damage the opponent, the amount of damage is indicated by injury = $y_{j}$.injury+1. The one who is injured wants to modify his place and attack other players from another place. This process expresses the exploitation of the algorithm which is simulated in equation (3).

(3) $$y_{inj.d}=y_{inj.d}+r\left(y_{b.d}-y_{inj.d}\right)$$

where, $y_{inj.d}$ represents the place of the injured player that is in dimension d, r indicates an amount between 0 and 1 which is selected at random. In a situation where the injured person can harm another player with a bullet, the $z_{j}$ value is considered zero. If the injured person is injured more than the defined limit, that person is considered dead. This is the state in the exploration algorithm. In this situation, the eliminated person may become visible in the continuation of the game and y_j.inj can be equal to 0. The number determined for the maximum number of injured is 3. Therefore, the algorithm does not get involved in early convergence and the exploration is performed well. An individual who becomes visible in the search space after dead is defined as equation (4):

(4) $$y_{inj.d}=r\times \left({ub}_{d}-{lb}_{d}\right)+{lb}_{d}$$

where, ${ub}_{d}$ and ${lb}_{d}$ represent the higher and lower ranges in solution space. The initial value of solution space is $\omega =\log_{10}\left(MaxCicle\right)$ which is become decreased based on the finest solution and is illustrated by $\omega =\omega +round\left(\frac{\omega }{2}\right)$. MaxCicle defines the max value of iteration. The renewed higher and lower ranges values are presented equation (5).:

(5) $${lb}_{d}=y_{b.d}-SD\left(\bar{y_{d}}\right)\;{ub}_{d}=y_{b.d}+SD\left(\bar{y_{d}}\right)$$

where, the finest solution discovered up to now in dimension d is indicated by $y_{b.d}$, the standard deviation of whole individuals is represented by $SD\left(\bar{z_{d}}\right)$. If the lower/higher range overreaches the main ${lb}_{d}/{ub}_{d}$, it adjusts to the main lower/higher ranges. The greatest individual in any iteration is maintained and supposed as an elite.

The maximum numeral of iterations, the numeral of individuals, and the dimensions of the problem determine the computational complexity of the defined algorithm. The complexity of calculation specifies through $O\left(m^{2}\right)$ and $O(n^{2}$) where n and m indicate the numeral of individuals and the numeral of iterations.

#### 2.2.3 Modified battle royal optimization algorithm

The Battle Royale optimization algorithm is a novel approach that offers good performance in solving some problems. But in solving some problems, there are weaknesses related to convergence and local optimization [21]. To improve the results obtained from the Battle Royale algorithm, two techniques are provided below. The initial modification is based on the OBL (Opposition-based learning) approach. According to the OBL approach, any formed solution candidate is assumed a pair of candidates, and the location of both candidates is complementary to each other. This concept is explained equation (6):

(6) $${\vec{y}}_{j}^{\text{new}}={\vec{y}}_{j}^{\max}+{\vec{y}}_{j}^{\min}-{\vec{y}}_{j}$$

where, ${\vec{y}}_{j}^{\text{new}}$ denotes the opposite location of ${\vec{y}}_{j}$, ${\vec{y}}_{j}^{\min}$ and ${\vec{y}}_{j}^{\max}$ stands for the minimum and maximum ranges of the solution. The appropriate solution of any novel pair candidate is stored and the other one is eliminated. In this paper, the initialization of 60 % population is obtained by chance and the remaining 40 % is obtained using the OBL approach. The second offered manner is chaos theory, in which quasi-random variables are formed instead of entirely random variables. Utilizing this technique raises the speed of meta-heuristic algorithm convergence. For this purpose, a sinusoidal map is employed. By renewing the r parameter in the above equation as a quasi-random variable, equation (7) is obtained:

(7) $$r_{1}\left(j+1\right)=P.r_{1}^{2}\left(j\right)\times \sin\left(\pi .r_{1}\left(j\right)\right)$$

where $r_{1}\left(j+1\right)$ defines the chaotic random value formed throughout the present iteration, and $r_{1}\left(j\right)$ stands for a chaotic value that formed at random in the former iteration. P indicates the control variable equal to 2.2 and $r_{1}\left(0\right)=0.6$.

The following Fig. 2 illustrates the flowchart related to the Modified Battle Royal optimization:

**Fig. 2:** Visual representation of the Modified Battle Royal optimization algorithm.

For delivering a suitable authentication to assess the efficiency of the offered Modified Battle Royal algorithm, the algorithm is executed to numerous standard benchmark functions and the comparison among the obtained outcome and the other three algorithms include the Multi-verse optimizer (MVO) [22], Owl Search Algorithm (OSA) [23], and Pigeon-inspired Optimization Algorithm (PIO) [24] is performed. The control parameters of the noted algorithms are listed in the following Table 1.

**Table 1:** Control parameters of the considered algorithms.

Algorithm	Parameter	Value
Multi-verse optimizer (MVO) [22]	$WEP_{\min}$	0.2
	$WEP_{\max}$	1
	Coefficient(P)	6
Owl Search Algorithm (OSA) [23]	$T_{dead}$	18
	|P|	10
	$Acc_{low}$	0.2
	$Acc_{high}$	1
Pigeon-inspired Optimization Algorithm (PIO) [24]	Number of Pigeons	200
	Space dimension	20
	Map and compass factor	0.2
	Map and compass operation limit	150
	Landmark operation limit	200
	Inertia factor (w)	1
	Self-confidence factor ($c_{1}$)	1.2
	Swarm confidence factor ($c_{2}$)	1.2

The details of the four utilized benchmark functions are illustrated in Table 2 below:

**Table 2:** Details of the utilized benchmark functions.

Formulation	Range	$F^{*}$
F1=x×sin(4x)+1.1y×sin(2y)	0<x, y<0	−18.55
$F2=0.5+\frac{\sin^{2}\left(\sqrt{x^{2}+y^{2}}-0.5\right)}{1+0.1\left(x^{2}+y^{2}\right)}$	0<x, y<2	0.5
$F3={\left|x\right|+\left|y\right|+\left(x^{2}+y^{2}\right)}^{0.25}\times \sin\left(30{\left({\left(x+0.5\right)}^{2}+y^{2}\right)}^{0.1}\right)$	[−∞,∞]	−0.25
$F4=10n+\sum_{i=1}^{n}\left(x_{i}^{2}-10\;\cos\left(2\pi x_{i}\right)\right),n=9$	[-5.12,5.12]	0

The individuals’ size is 50 and the max number of iterations throughout the optimization approach is 200. All mentioned functions have been executed 40 times independently. Consequently, the min value, max value, average value, and Std (standard deviation) of the benchmark functions have been used as the measurement indicators. In the following Table 3, the numerical attainments of the optimizers employed for the analyzed benchmark functions are listed.

**Table 3:** Numerical attainments of the utilized optimizers.

Function	Indicator	Algorithm			
		MVO [22]	OSA [23]	PIO [24]	MBRO
$F_{1}$	Max	−9.343	−12.123	−16.152	−18.75
	Min	−13.398	−14.398	−14.52	−14.44
	Median	−11.364	−13.669	−15.27	−15.65
	Std	4.244	3.948	3.25	2.45
$F_{2}$	Max	0.758	0.748	0.436	0.426
	Min	0.564	0.538	0.524	0.511
	Median	0.661	0.648	0.591	0.587
	Std	0.049	0.023	0.004	0.002
$F_{3}$	Max	−0.091	−0.298	−0.324	−0.332
	Min	−0.321	−0.345	−0.357	−0.389
	Median	−0.260	−0.275	−0.321	−0.374
	Std	0.245	0.219	0.019	0.012
$F_{4}$	Max	13.474	11.548	8.365	3.482
	Min	1.705	1.018	0.009	0.002
	Median	7.698	6.832	4.745	1.298
	Std	5.345	5.165	2.483	1.173

The results demonstrate that the efficiency of the four optimization algorithms varies depending on the benchmark function being analyzed. For example, in the case of function $F_{1}$, MBRO outperforms the other algorithms in terms of the maximum, minimum, median, and standard deviation of the attained values. Similarly, for function $F_{4}$, MBRO outperforms the other algorithms in terms of the maximum and median attained values, but its standard deviation is higher than that of MVO and OSA. On the other hand, for function $F_{2}$, MBRO performs similarly to the other algorithms in terms of the maximum, minimum, and median attained values, but its standard deviation is slightly higher than that of the other algorithms. For function $F_{3}$, MBRO performs worse than the other algorithms in terms of the maximum, minimum, and median attained values, but its standard deviation is lower than that of MVO and OSA.

The results generally suggested that MBRO is a competitive optimization algorithm that can achieve good performance on certain benchmark functions. However, its efficiency can vary depending on the specific function being analyzed. The comparison with other popular optimization algorithms in the literature such as MVO, OSA, and PIO provides a useful benchmark for evaluating the performance of MBRO. By analyzing the numeric attainments of the different algorithms across the benchmark functions, researchers can gain insights into the relative strengths and weaknesses of each algorithm.

It is important to note that the results presented in Table 3 are only a sample of the benchmark functions that were analyzed. To draw more robust conclusions about the efficiency of the different optimization algorithms, it would be necessary to analyze a larger set of benchmark functions and perform statistical tests to assess the significance of the differences in performance between the algorithms.

### 2.3 The proposed network

In this section, we will go over the overall structure of the sports image classification approach created. Fig. (3) shows the graphical abstract of the proposed network.

**Fig. 3:** Graphical abstract of the proposed network.

#### 2.3.1 Feature extraction by MobileNetV3 model

This section describes how to use a method to fine-adjusting of the feature extraction phase and the MobileNetV3. The main purpose is to obtain pertinent image embeddings using a pre-trained model on various sports image datasets.

In this phase, the extracted image embedding is given to the feature selection stage which follows. Compared to past studies, this feature selection uses a new modified battle royal optimization algorithm to improve recognition accuracy, choose only necessary features, and shrink the feature representation space of the entire suggested outline.

MobileNetV3 is an ideal model to carry out image recognition, providing a core feature in the extraction stage [25,26]. To avoid having to build the model from the ground up and accelerate the learning process, a MobileNetV3-Large pre-trained model was taken from the ImageNet dataset and tailored to recognize sports through transfer learning and fine-adjusting.

By applying the standard procedure, the MobileNetV3 model has been fine-adjusted and successfully extracted the necessary image embeddings. To do this, the top two of the MobileNetV3 output layers utilized for image classification with a 1 × 1 point-wise convolution have been replaced to maximize image features. This 1 × 1 point-wise convolution can work as an MLP (multi-layer perceptron) to not only perform image classification but also reduce dimensionality by integrating various nonlinearity operations.

Furthermore, to enhance the model's accuracy and performance on various datasets related to the classification task, extra 1 × 1 point-wise convolutions have been implemented. After fine-adjusting, the output of the 1 × 1 point-wise convolution is flattened to generate a 128-size image embedding for each image in the dataset. Finally, these extracted image embeddings are used for feature selection.

The modified MobileNetV3 configuration, presented in Fig. (4), is a highly efficient platform for extracting features from sports images. To further refine the model and achieve optimal results, we fine-adjusted it for 200 epochs with 15 different random runs. A batch size of 32 with a stochastic gradient descent approach called RMSprop is employed with a learning rate of 1e-4 to perform the fine-adjusting. This method yielded the highest classification accuracy on each dataset.

**Fig. 4:** The modified MobileNetV3 configuration.

To reduce overfitting and increase the model's ability to generalize, data augmentation was utilized during the preprocessing stage. This method included transformations such as random horizontal flip, random vertical flip, and random crop. The size of input images is transformed to 224 × 224 because of the nature of the network.

#### 2.3.2 Feature selection based on binary modified battle royal optimization algorithm

The modified battle royal optimization algorithm is adapted to work as a feature selection method in its binary form, as shown in Fig. (5). This adaptation makes the modified battle royal optimization algorithm suitable for dealing with discrete problems since its original version was only designed to handle real-valued problems. The modified battle royal optimization algorithm consists uses the following technique to provide binary output:

**Fig. 5:** Example extracted images from the datasets for the analyzed sports groups.

By assuming $x_{i}$ as the solution candidates, the binary output can be achieved by equation (8):

(8) $$x_{i}^{b}=\left\{ \begin{array}{c} 1,if\;x_{ij}>1/2\\ 0,otherwise \end{array}\right.$$

Leveraging the powerful features of the optimal solution $x^{b}$, we can effectively narrow down our testing set for the SVM classifier. Subsequently, by utilizing various performance measures, we will be able to accurately assess the predicted output.

## 3 Results and discussions

### 3.1 System configuration

The datasets utilized in the sports image classification challenge are discussed in this part, as well as the distribution of the related samples. In our tests, the network was trained and tuned using a common dataset. A thorough explanation of the dataset is provided in the section that follows. On a machine with an Intel® Core™ i7 CPU working at 2.5 GHz, speeds of 2.00 GHz, 16 GB of memory, and a 64-bit operating system, the proposed structure is put into practice.

For the categorization of sports images, a hybrid technique based on MobileNetV3 and a modified battle royal optimization algorithm was developed. The intended classification for the investigation was coded in the MATLAB R2019b framework, and the outcomes were cross-referenced with a database.

### 3.2 Dataset description

The images used for analysis are 240 × 320 pixels in size. There is a variety of image characteristics in each category; some of the images are blurry, some are dark, and others are clear. Furthermore, these images are from disparate sources, so the background and camera angles are not similar. This makes analysis onerous. Our dataset is a tough yet optimal choice for investigation due to the varying backgrounds, the camera views, and the blurriness of the photographs. An example of these different picture types is presented in Fig. (5).

A dataset containing 7500 frames has been generated by downloading videos from YouTube belonging to various sports categories, such as including Rugby [27], Cricket [28], Volleyball [29], Badminton [30], Tennis [31], and Basketball [32], and then extracting frames from the movies. 25 % of the data has been leveraged for testing with the remaining 75 % used for training purposes, following the usual classification standard. Table 4 offers a comprehensive statistical breakdown of the images employed for sport-specific training and testing. The table is organized into three columns: the first column indicates the sport category, the second column indicates the total number of images utilized for each sport, and the third and fourth columns indicate the number of images used for training and testing, respectively.

**Table 4:** Statistical breakdown of the images utilized for various sports-related training and test.

Sport Category	Total Images	Training Data	Testing Data
Rugby	1910	1300	610
Crocket	1578	1150	428
Badminton	1823	1315	508
Basketball	1840	1320	520
Tennis	1795	1300	495
Volleyball	1780	1280	500
Total	10726	7665	3061

The results presented in Table 4 provide valuable information about the data used for training and testing in the sports-related classification tasks. The table shows that a total of 10,726 images were utilized, with the majority of images used for training (7665 images) and the remaining images used for testing (3061 images). The table also shows that the number of images utilized for each sport category varied, with Rugby having the highest number of images (1,910) and Croquet having the lowest number of images (1,578). The breakdown of images into training and testing sets also varied by sport, with Badminton having the highest number of images used for training (1,315) and Volleyball having the highest number of images used for testing (500).

The data is classified using neural networks, and its accuracy is 97.40 %. To evaluate the effectiveness of our training, the dataset is trained using different classifiers such as the Convolutional neural network (CNN) [3], Bayesian classifier [8], and InceptionV3 [2]. The confusion matrix for neural networks is shown in Table 5.

**Table 5:** Confusion results of the comparative models.

	Badminton	Basketball	Crocket	Rugby	Tennis	Volleyball	Σ
Badminton	494	0	0	0	0	0	610
Basketball	0	520	0	0	0	0	520
Tennis	10	0	0	10	480	0	495
Rugby	0	0	20	590	0	0	610
Crocket	0	0	415	13	0	0	428
Volleyball	0	0	0	0	10	490	500
Σ	504	520	535	613	490	490	3163

The cells in the table contain the count values representing the number of predictions made by the model. Let's break down the provided confusion matrix: The sports classes considered in this classification task are: Badminton, Basketball, Crocket, Rugby, Tennis, and Volleyball. The first row represents the predictions made for the Badminton class. It shows that out of a total of 610 instances of Badminton, the model correctly predicted 494 instances as Badminton, while it made incorrect predictions for the remaining instances of Badminton. Similarly, the second row represents the predictions made for the Basketball class. The model correctly predicted 520 instances as Basketball out of a total of 520 instances in the dataset. The third row corresponds to the Tennis class. The model correctly predicted 480 instances as Tennis, but it misclassified 15 instances as Crocket and 10 instances as Rugby. The fourth row represents the Rugby class. The model correctly predicted 590 instances as Rugby, but it misclassified 20 instances as Crocket. The fifth row corresponds to the Crocket class. The model correctly predicted 415 instances as Crocket, but it misclassified 13 instances as Tennis. The sixth row represents the Volleyball class. The model correctly predicted 490 instances as Volleyball out of a total of 500 instances. The last row provides the totals for each column, indicating the actual number of instances for each class.

Because our dataset is novel and no prior study has been done on it, we compared the results of our recommended framework with those from findings from other classifiers. Table 6 compares the findings.

**Table 6:** Simulation results for comparing the methods.

Sport Category	InceptionV3 [2]	Bayesian classifier [8]	CNN [3]	Proposed method
Volleyball	97.45 %	97.84 %	98.05 %	99.17 %
Basketball	93.44 %	96.80 %	91.87 %	98.8 %
Badminton	97.13 %	70.29 %	98.61 %	99.62 %
Rugby	78.29 %	99.37 %	95.08 %	95.11 %
Tennis	98.16 %	99.14 %	96.62 %	99.64 %
Cricket	84.34 %	97.61 %	86.14 %	97.04 %
Total %	91.46 %	92.27 %	94.89 %	97.40 %

Table 6 shows the results of a simulation comparing different methods for classification in various sports categories. The four methods being compared are InceptionV3, the Bayesian classifier, CNN, and the proposed method. In general, the proposed method outperforms all other methods across all sports categories, achieving an average accuracy of 97.40 %. Specifically, it achieves particularly high accuracy rates in volleyball (99.17 %), badminton (99.62 %), and tennis (99.64 %). The second-best performing method is the CNN with an average accuracy rate of 94.89 %, which performs well in basketball and rugby but not as well in cricket. The InceptionV3 model has an overall lower accuracy rate at 91.46 % but still performs relatively well in some sports such as volleyball and tennis. The Bayesian classifier performed worst among all models with an average accuracy rate of only 92.27 %. These findings suggest that the proposed method can be highly effective for classifying images related to various types of sports activities by using deep learning techniques such as Convolutional Neural Networks (CNNs). This could have significant practical applications for tasks like automated video analysis or surveillance systems aimed at detecting specific sporting events or activities from live feeds or recorded footage.

## 4 Conclusions

The media's coverage of sports has increased dramatically, and with that growth has come a greater requirement for the correct classification of sports photographs. The human curation of characteristics used in traditional approaches makes them unsuitable for managing enormous amounts of data and separating pictures that resemble one another closely. The purpose of this work was to accelerate automatic sports image classification using sizable data sets by utilizing deep learning. For this, a framework that combines the MobileNetV3 model with a modified battle royale optimization method was created. The proposed model was then applied to different images gathered from the internet and the results were compared with some other state-of-the-art methods, including InceptionV3, Bayesian classifier, and convolutional neural network. The results indicated that the proposed method outperformed all other methods across all sports categories, achieving an average accuracy of 97.40 %. Specifically, it achieves particularly high accuracy rates in volleyball (99.17 %), badminton (99.62 %), and tennis (99.64 %). By using this architecture to already successfully identify sports activities, the method can be utilized to generate a dataset specifically for sports, demonstrating the effectiveness of the approach. By including temporal information, the framework may be used for activity analysis and video searches.

## Data availability statement

The authors are unable or have chosen not to specify which data has been used.

## CRediT authorship contribution statement

**Bing Wang:** Conceptualization, Data curation, Formal analysis, Software, Supervision, Visualization, Writing – review & editing. **Asad Rezaei sofla:** Conceptualization, Data curation, Formal analysis, Methodology, Resources, Visualization, Writing – original draft, Writing – review & editing.

## Declaration of competing interest

The authors declare that they have no known competing financial interests or personal relationships that could have appeared to influence the work reported in this paper.
